This article has been retracted.

# Analysis of Clinicopathological Factors Associated with Radiation-Induced Cystitis in Patients with Cervical Cancer

**DOI:** 10.1155/2022/6216072

**Published:** 2022-04-15

**Authors:** Ling He, Zhenyu Wang, Jianhui Chen, Ling Chen, Peijuan Chen, Wenzhi Cai

**Affiliations:** ^1^Shenzhen Hospital of Southern Medical University, Shenzhen, Guangdong 518101, China; ^2^Department of Radiation Oncology, Nanfang Hospital of Southern Medical University, Guangzhou, Guangdong 510515, China; ^3^Department of Radiation Oncology the First Affiliated Hospital, The Sun Yat-sen University, Guangzhou 510080, China; ^4^Department of Rheumatology, Nanfang Hospital of Southern Medical University, Guangzhou, Guangdong 510515, China

## Abstract

**Objective:**

To analyze the clinicopathological characteristics associated with radiation-induced cystitis (RIC) in patients with cervical cancer treated with chemoradiotherapy (CRT) alone or postoperational (post-op) CRT.

**Methods:**

107 patients with cervical cancer were retrospectively recruited into the study. The surgical status, FIGO staging, total and fractionated doses of radiotherapy (RT), and multiparameters including the dose, volume irradiated to the total bladder, and bladder wall were evaluated for RIC. The criteria on RIC were referred to CTCAE v5.0.

**Results:**

Surgical operation and post-op CRT were delivered in 65 patients and CRT or RT alone in 42 patients. Among those with post-op CRT, 33/34 (97.06%), 22/43 (51.16%), and 10/30 (33.33%) patients were classified as FIGO stage I, II, and III/IV, respectively. The incidence of RIC was 30.84% for the whole group with 87.87% occurred in stage I and II patients. The incidence of CTCAE grade 2 and beyond was significantly higher in patients treated with post-op CRT than those with CRT alone (13.85% vs 2.38%, *p* = 0.043). Further analyses showed that the CTCAE level of RIC in the post-op CRT group was related to the relatively smaller average bladder volume (*p* = 0.029), whereas the difference in volume of bladder and bladder wall irradiated to 35.0 Gy or 40.0 Gy was not statistically significant between patients with or without RIC. Conclusion. The combination of surgery and post-op CRT may increase the incidence and severity of radiation-induced cystitis when compared to CRT alone, suggesting that bladder dysfunction associated with surgical procedure might increase the frequency and severity radiation related bladder toxicity. Further study is merited.

## 1. Introduction

Radiotherapy is an important part of the comprehensive treatment of cervical cancer. It has been estimated that approximately 60% to 70% of cervical cancer patients receive radiotherapy alone or in combination with chemotherapy. In addition to the target area during radiotherapy, the normal tissues adjacent to the cervix, i.e., colon and rectus, small intestine, bladder, urinary tract, female reproductive organs, bone, and skin, will also be exposed to varying volume and dose of irradiation with certain degree of radiation-induced damage. The degree of radiation damage mainly depends on the total and fractionated doses of radiotherapy, the volume of normal organs exposed to irradiation, the radiation technique applied, patient factors including chronic medical conditions, and other related factors such as surgical operation. [1–3]. Radiotherapy-associated complications on the bladder are mainly radiation-induced cystitis (RIC) with clinical symptoms and signs of frequent urination, urgency, dysuria, and hematuria. Intractable arterial hemorrhage may also occur in patient presented with severe complication [2, 4–7]. It has been observed that 50% ∼ 60% of patients will begin to present symptoms and signs of RIC of varying degree within 3 to 4 weeks at the initiation of pelvic irradiation which may persist for a long period of time [4, 8].

As advancement in radiotherapy technology and application of intensity modulated radiotherapy (IMRT) and volumetric intensity modulated arc radiotherapy (VMAT), the dose conformity of the cervical cancer target area has significantly been improved with significant reduction of the exposure dose to the surrounding normal tissues; hence, radiation-associated incidence and severity of proctitis and cystitis have been greatly reduced [9, 10].

With the advancement of surgical technology, total hysterectomy combined with bilateral adnexectomy resection and pelvic lymph node dissection for early cervical cancer has been reported to achieve the same curative effect as RT and chemotherapy [11] and thus recommended as the standard of care by National Comprehensive Cancer Network (NCCN) [12]. Post-op RT combined with chemotherapy has been recommended for the patients with positive resection margins, cancer invasion to the region of the parauterine (s), pathological adenopathy, and infiltration into the deep cervical muscle to reduce the risk of loco-regional recurrence [13]. During the surgical procedure, the bladder autonomic nerve may be partially destroyed causing the characteristics of the elastic muscle fibers of the bladder wall to decrease which leads to neurogenic bladder dysfunction presenting with frequent urination, urgency, and the occurrence of lower urinary tract symptoms such as urinary incontinence [14, 15].

It has been reported that the occurrence of RIC is not only related to the total and fractionated doses of RT, the volume and dose of bladder exposed, changes of bladder filling, the individualized bladder sensitivity of patients, and other complex factors [16–21]. The autonomic nerve related to the bladder might be completely or partially destroyed in the process of surgery, which has been studied in patients with prostate cancer [22–24]. There are few studies on the factors related to the occurrence of RIC after adjuvant radiotherapy/chemotherapy after cervical cancer surgery. Change in the degree of bladder filling has been reported to influence the position and wall thickness of the bladder and have a greater impact on the precision of RT to the targeted region and its surrounding normal tissues [25, 26]. There has been extensive research on the radiation associated toxicity on the rectal wall with the establishment of predictive model in cervical cancer patients [27]. Whereas the research on the radiation associated toxicity on the bladder especially for patients with post-op CRT has rarely been reported.

This study is designed to analyze the clinicopathological characteristics and volumetric dosimetry parameters in patients with cervical cancer treated with CRT alone or post-op CRT associated with RIC in order to explore potential measures to reduce the incidence of RIC and improve the quality of life.

## 2. Materials and Methods

### 2.1. Clinical Data

This study has been approved by the Medical Ethics of Investigation Research Board of the Institute (NFEC-2022-023). A total of 107 patients with cervical cancer were recruited who underwent CRT alone or in combination with surgical operation from January 2017 to December 2018. All patients underwent physical examination and CT imaging studies of the chest, abdomen, and pelvis prior to treatment; among them, some underwent pelvic MRI and 11 (10.3%) received F18-FDG PET-CT scan, using the International Federation of Gynecology and Obstetrics (FIGO) criteria as clinical staging.

Criteria for the case inclusion: (1) Pathological diagnosis as cervical squamous cell carcinoma prior to treatment, (2) locally or locally advanced cervical cancer with no evidence of distant metastasis by multiple imaging studies prior to treatment, and (3) complete clinicopathological data. Criteria for the case exclusion: (1) Patients with distant metastases were excluded by multiple imaging studies prior to treatment, (2) patients with other malignant tumors, (3) patients with a history of pelvic radiotherapy and chemotherapy, and (4) loss to follow-up.

### 2.2. Surgical Operation

The surgical procedures for cervical cancer include total hysterectomy and bilateral adnexectomy combined with pelvic lymph node dissection. The patients will be referred to receive post-op CRT when the pathological diagnosis shows sign(s) of risk(s) of recurrence, i.e., large primary tumor, deep cervical myometrial invasion, positive surgical margin(s), parametrial invasion, positive lymphadenopathy, and other risk factors.

### 2.3. Procedure for Radiotherapy

The patient was immobilized in the supine position on the homemade vacuum bag for CT simulation with Big Bore CT scanner (Brilliance Big Bore, Philips). Prior to simulation, the patient was instructed to empty the bladder and then drink approximately 300 ml of water mixed with the contrast agent, iopamidol (Producer, Country). Based on the diagnosis with CT, reference points (0°, 90°, and 270°) were marked on the positioning film with crosses after laser alignment, as close to the surface corresponding to the target area. The plain and contrast-enhanced planning CT scans with 3.0 mm of thickness were obtained accordingly using spiral CT scanner with the scan range extended from the inferior aspect of L1 to 5 cm below the lower edge of the obturator while the images were constructed and then imported to the treatment planning system (TPS) station for target delineation.

### 2.4. Target Delineation, Radiotherapy Plan Design, and Evaluation

Target volume was defined according to the recommendations of the International Commission on Radiation Units and Measurements (ICRU) reports No. 50 and 62 and Myerson RJ et al. [28, 29]. The primary gross tumor volume (GTVp) was delineated further according to the information obtained from the diagnostic CT and F18-FDG PET-CT, including the primary tumor of the cervical area and local tumor infiltration or postoperative tumor bed area; suspected positive lymph nodes according to image data are defined as GTVn. The clinical target volume (CTV1) was the subclinical lesion with potential metastasis. PGTVp, PGTVn, and PTV1 were obtained by adding uniform margins 0.6 cm to GTVp, GTVn, and CTV1, respectively. The organs at risk (OAR) volumes were outlined in the small bowel, the rectum, the colon, the marrow, the kidneys, the bladder, the femoral heads, and the spinal cord.

Delineation of the bladder wall: the bladder wall structure is generated by shrinking the outline of the bladder by the thickness of the bladder wall. The relationship between the bladder wall thickness T_BW_ and the bladder volume *V*_B_ is based on the experience reported in the literature [30–32]: T_BW_ = EXP (3.355–0.484*V*_B_).

All patients received 5–9 fields intensity-modulated radiotherapy. IMRT plans were performed using the inverse planning system (Monaco, version 2.0, Sweden). All plans were delivered using 6 MV photons, Elekta ELE-2775. IMRT plans were generated using 5–9 coplanar equi-spaced fields with static multileaf collimator. The isocenter was placed at the geometric center of the PTV1. The IMRT treatment plans were designed to deliver in a single-phase process (with simultaneously integrated boost, SIB); a dose of 45–50 Gy to the PTV1 in 25 fractions (1.8–2.0 Gy daily fractions) and 60 Gy to the parauterine ligament of PGTVp and PGTVn (2.4 Gy daily fractions) over the period of 5 weeks. 50 Gy in 25 fractions was delivered to the uterine while 30 Gy of brachytherapy would be added in 5–6 fractions for patients with CRT alone. Planning objectives for OARs were defined as follows: small bowel: *D*_5_ ≤ 50 Gy, *D*_max_ ≤ 55 Gy; rectum: V_55Gy_ ≤ 5%, *D*_max_ ≤ 60 Gy; colon: *D*_max_ ≤ 60 Gy; marrow: V_20Gy_ ≤ 50%; kidneys: *D*_mean_ ≤ 15 Gy, V_18Gy_ ≤ 30%; bladder: V_50Gy_ ≤ 30%, *D*_max_ ≤ 65 Gy; femoral heads: *D*_5_ ≤ 45 Gy; and spinal cord: *D*_max_ ≤ 45 Gy. The requirements of evaluating radiotherapy plan include 95% of the prescribed dose (*D*_95_) covers at least 95% of the target volume (V_95_). It is completed and confirmed by senior radiotherapy physicians and physicists before being executed on the machine.

### 2.5. Data Collection and Follow-Up

The median follow-up time was 9 months (4–16 months). Collect the patient's age, stage, chemotherapy regimen and cycle, smoking history, diabetes history, total radiation dose and fractional dose, CTV volume, bladder volume, bladder wall volume, and bladder and bladder wall dose volume parameters such as D_mean_, *D*_max_, V_35_, and V_45_.

The follow-up is mainly through inquiries about hospitalized medical records and telephone follow-up, recording the patient's survival, death or loss to follow-up status, and urinary system reactions caused by external irradiation.

### 2.6. Evaluation Criteria for Radiotherapy Response

The grading standard of urinary system toxicity and side effects refers to the evaluation standard of common adverse events (CTCAE) *V*5.0 [33, 34]: Grade 0: no radiotherapy reaction; Grade 1: microscopic hematuria, mildly increased urinary frequency, urgency, dysuria, nocturia, and urinary incontinence; Grade 2: moderate hematuria; moderate increased urinary frequency, urgency, difficulty urinating, nocturia, and urinary incontinence; need catheter and bladder irrigation; and affect instrumental activities of daily living; Grade 3: massive hematuria; need blood transfusion, intravenous infusion of drugs, and hospitalization; and need elective invasive treatment; Grade 4: life-threatening; urgent invasive treatment is required; and Grade 5: death due to RIC.

The score of toxicity scores were evaluated during the period of treatment or by follow-up. The time of follow-up ranges from 6 to 30 months after radiotherapy. Due to the incomplete after loading brachytherapy data of some patients, this study was focused on the investigation of clinicopathological impacts on urinary system toxicity caused by external radiation therapy.

### 2.7. Statistical Methods

All data were analyzed using SPSS 23.0 statistical software. Measurement data are expressed by mean standard deviation, the independent sample *t* test is used for comparison between groups, and the chi-square test is used for comparison between count data. *p* < 0.05 is considered statistically significant.

## 3. Result

### 3.1. Comprehensive Treatment of Cervical Cancer Patients of Different Stages

There were 107 patients with the median age of 53 years old ranging from 28 to 71 years. According to the FIGO staging, the number of stages I, II, III, and IV cases were 34, 43, 25, and 5, respectively. 60.7% (65/107) of patients underwent total hysterectomy with bilateral appendage resection. 96.3% (103/107) of patients received combination of radiotherapy and chemotherapy. The regimen for chemotherapy is TP/TC (Taxotere + cisplatin/nedaplatin), and concurrent chemotherapy with DDP (platinum) is used as sensitization during radiotherapy. Detailed clinicopathological characteristics are presented in Table 1.

Radiotherapy alone or concurrent with chemotherapy was delivered in 1, 21, and 20 patients in stage I, stage II, and stage III/IV, respectively, while post-op CRT was administered in 33, 22, and 10 patients in stage I, stage II, and stage III/IV, respectively.  Figure 1 shows the representative dose profiles of bladder in different filling states, underfilling, properly filling, or overfilling dose profiles of three different bladder filling states.

No bladder toxicity was observed in 74 patients (69.2%) who were treated with CRT or in combination with surgical procedure. The incidence for patients with grades 1, 2, and 3 RIC was 21.5% (23/107), 4.7% (5/107), and 4.7% (5/107), respectively. No patient was observed to manifest RIC of grade 4 or above.

The association of incidence of RIC in accordance with the FIGO stage and dosimetric parameters is presented in Table 2. We observed that the prescribed dose and fractionated dose increased accordingly with the increase of FIGO stage, especially significant increment in patients in stages III and IV (*p* < 0.001). The bladder was exposed to the higher maximum dose of the irradiation in locally advanced cases (*p* < 0.05), whereas no significant difference was observed in the average dose. With the expansion of tumor invasion, the volume of CTV in the subclinical target area of potential metastasis also increased (*p* < 0.05) and the chemotherapy cycle increased, but there was no statistical difference. There was no significant difference in bladder volume and bladder wall volume in patients of different stages (*p* > 0.05).

The combination of operational procedure and CRT was administered in 33/34 (97.06%), 22/43 (51.16%), and 10/30 (33.33%) patients for FIGO stages I, II, and III/IV, respectively. The incidence of RIC was 30.84% for the whole group. The number of cases of RIC in patients with stages I, II, and III/IV cervical cancer was 12 (35.29%), 17 (39.53%), and 4 (13.33%), respectively.

### 3.2. Relationship between Surgery and Adverse Bladder Reactions

The treatment for patients with early-stage cervical cancer is mainly surgery and post-op CRT while those with the locally advanced with concurrent is CRT. In this study, 65 patients underwent surgical operation including total hysterectomy and bilateral adnexectomy combined with pelvic lymph node dissection. Among those with post-op CRT, 33/34 (97.06%), 22/43 (51.16%), and 10/30 (33.33%) patients were classified as FIGO stages I, II, and III/IV, respectively. The incidence of RIC was 30.84% for the whole group.

Table 3 presents the association of CTCAE and parameters of CRT in cervical cancer patients between groups of post-op CRT and CRT alone. Among them, 9 cases (13.85%) in the group of post-op CRT developed RIC with CTCAE grade 2 or higher while only one patient (2.38%) in the group of CRT alone had only CTCAE grade 2 or higher, and the difference in RIC grade 2 or higher was statistically significant (*p* = 0.043).

The difference of CTCAE grades in bladder volume between the groups of post-op CRT and CRT alone is shown in Figure 2. The CTCAE levels of patients undergoing surgery and post-op CRT manifested an inverse relationship with their bladder volume, i.e., the smaller the bladder volume, the more severe the bladder dysfunction. The average bladder volume for those with CTCAE grade 3 symptoms or without was 368.90 cm^3^ and 186.60 cm^3^ (*p* = 0.029), respectively, whereas there was no correlation between CTCAE and bladder volume in the CRT group alone.

### 3.3. Relationship between Dosimetry Parameters and RIC

The patients were subgrouped according to the bladder toxicity of different CTCAE grades. The age, stage, chemotherapy cycle, CTV volume, bladder volume, bladder wall volume, and bladder were analyzed according to CTCAE grades ranging from 0 and 3. There was no statistical difference in the average dose, prescribed dose, single dose, and maximum bladder dose. The volume of bladder exposed to radiation 35 Gy or 40 Gy (V_35_ and V_40_) was observed to decrease as the severity of RIC increased.

Figure 3(a) shows the bladder and bladder wall volume distribution of 107 cervical cancer cases with different CTCAE grades. The volume of bladder was 335.50 cm^3^ (28.44 ∼ 797.88 cm^3^), 301.77 cm^3^ (53.43 ∼ 543.92) cm^3^, 219.19 (92.61 ∼ 320.81) cm^3^, and 205.40 cm^3^ (37.69 ∼ 435.43 cm^3^) for patients with CTCAE level 0, 1, 2, and 3 groups, respectively. The volume of bladder wall was 61.67 cm^3^ (27.27 ∼ 100.46 cm^3^), 57.16 cm^3^ (29.42 ∼ 80.56 cm^3^), 55.66 cm^3^ (36.60 ∼ 67.01 cm^3^), and 46.49 cm^3^ (28.64 ∼ 71.37 cm^3^) for patients with CTCAE level 0, 1, 2, and 3 groups, respectively. Further analyses showed that the patients who presented with more severe RIC seemed smaller volume of bladder, especially for those experienced surgical procedure.

Figure 3(b) shows the relationship between the distribution of the volume of 35 Gy or 40 Gy of bladder and bladder wall and different grades of RIC in 77 cases of stage I and II cervical cancer. The changes of bladder V_35_ and V_40_ are similar to those in Figure 3(a). The data show that patients with smaller bladder volume, V_35_ and V_40_, present more severe RIC; the smaller the bladder volume, the thicker the bladder wall.

As presented in Table 2, the occurrence of RIC is mainly concentrated on the cases of stages I and II cervical cancer accounting for 87.87%. Further analyses demonstrated that the occurrence of RIC of different levels, such as age, surgery, chemotherapy, prescription dose, single dose, and CTV volume, are not significantly different as presented in Table 4. The volume of bladder and bladder wall tends to decrease with the aggravation of toxicity of RIC, to the V_35_ and V_40_, which the difference is statistically significant. It is consistent with the total prescription dose, and the average dose has no difference. Whereas there is no significant difference in the dosimetric parameters such as *D*_max_ and D_mean_ exposed to the bladder or bladder wall.

## 4. Discussion

With the introduction of IMRT technique, the incidence of radiation associated toxicity including RIC has been significantly reduced [35]. Our research has shown that the incidence of CTCAE grade 2 and beyond was 2.38% in patients treated with CRT alone, which was significantly lower than those treated with post-op CRT (13.85%). The CTCAE level of RIC in the surgery and the post-op CRT group was related to the relatively smaller average bladder volume, whereas the difference in volume of bladder and bladder wall irradiated to 35.0 Gy or 40.0 Gy in patients with stages I and II cervical cancer was not statistically significant between patients with or without RIC. Our data suggest that the combination of surgical procedure and post-op CRT may increase the incidence and severity of radiation-induced cystitis when compared to CRT alone indicating that the neurogenic bladder associated with surgical procedure might be one of the main causes of radiation-related bladder toxicity.

The variation in position and/or volume of the organs, i.e., bladder, intestine, and rectum, are frequently observed during the period of radiotherapy of cervical cancer, which may affect the accurate administration of radiotherapy and lead to over dose of irradiation to the adjacent normal tissues. Among them, the bladder volume changes most obviously with the degree of holding urine. It is of clinical significance to precisely deliver each fractionation of radiotherapy during treatment since the difference in bladder volume will affect the precision of formulation of radiation treatment plans and delivery of radiotherapy as shown in Figure 1. When the bladder volume is too small (<100 ml) due to insufficient urination in CT simulation image, the CTV coverage would be extended to the surrounding normal tissues, including bladder detrusor, sphincter, and peripheral nerves. During the implementation of radiotherapy, these organs and nerves are inevitably exposed to higher doses. In the case of moderate holding of urine, the bladder volume is about 250∼400 ml, and the anterior, the top, and lateral of the bladder are stretched well to keep it away from the high-dose irradiation area; thus, to keep the bladder full during the implementation of radiotherapy, consistency is conducive to improving the local control rate and reducing the bladder, rectum, and small bowel radiotherapy response. Although overfilling of the bladder shows a lower dose to the normal organ dose in the radiotherapy plan design, it is difficult to keep the bladder of similar retention volume at each fractionation during the period of actual treatment lasting more than a month leading to relatively large deviation of the dose distribution is relatively large. There have been reports that support this view [26, 36].

There have been reported favorable long-term survival and less toxicities of bladder, rectum, and sexual function in patients with prostate cancer. Robinson et al reported their meta-analysis by comparing the rates of erectile function after RT, radical prostatectomy with or without preservation of autonomous nerve and cryosurgery. The rate of impotency was 40%, 66%, 75%, and 87% for RT, nerve-sparing radical prostatectomy, nonnerve sparing radical prostatectomy, and cryosurgery [37].

Approximately 60% of the patients in this study underwent extensive total hysterectomy and bilateral adnexectomy combined with pelvic lymph node dissection which may achieve the same curative effect as radiotherapy and chemotherapy in patients with early cervical cancer. There have been many studies of the dysfunction on autonomic nerve in patients with cervical cancer who were treated with surgery and post-op CRT [38]. Whereas there has been extensive research on the autonomic nerve related to the sexual bladder dysfunction might be completely or partially destroyed in the process of surgery in patients with prostate cancer [39–41].

This study shows that stages Ib ∼ IIa patients were mainly received surgical operation followed by post-op CRT, while stages III and IV patients mainly receive concurrent radiotherapy and chemotherapy; the incidence and severity of RIC in the post-op CRT group is higher than that in the radiotherapy group. Our study showed that the incidence of CTCAE grade 2 and beyond was 2.38% in patients treated with CRT alone, which was significantly lower than those treated with post-op CRT (13.85%). As the pathological stage increases and patients in advanced stage are often accompanied by lymph node metastasis, the prescribed total and fractionated dose to the lymph drainage is also correspondingly increased, the radiotherapy target area will be larger. This study also showed the similar trend according to the pathological stage, but the toxicity of the bladder did not show a trend of increasing with the advancement of the pathological stage, which might benefit from the application of IMRT technique.

The existing dose evaluation parameters are also summarized by many international medical institutions through years of clinical experience needed to be evaluated accordingly with clinical outcomes [42]. In the clinical practice, several measures have been adopted to ensure the accurate implementation during the process of radiotherapy, i.e., more effective position fixation apparatus, image guidance technology, and bladder measurement measures [43], whereas it is still difficult to ensure the patient's relatively constant position of bladder given the variation of volume and bladder wall at the time of simulating and optimizing the plan of radiotherapy through implementing its delivery. Therefore, the actual absorbed dose to the bladder and bladder wall cannot be monitored for every individual delivery of radiotherapy.

This study is a retrospective research that did not analyze the effect of brachytherapy on the severity of RIC, whereas brachytherapy is mainly applied for those with locally advanced cervical cancer who were treated by radiotherapy with or without chemotherapy. Therefore, the toxic and side effects of patients who were exposed to bladder radiation after brachytherapy were not studied. During the follow-up, patients were specifically enquired about their lower urinary tract symptoms before brachytherapy. Nevertheless, it is not ruled out that some patients could not distinguish whether they had frequent and urgent urination before brachytherapy.

## 5. Conclusion

In summary, surgical operation and post-op CRT was mainly administered for patients with early cervical cancer and CRT alone for those with locally advanced disease. The combined treatment modalities may increase the incidence and severity of radiation-induced cystitis when compared to CRT alone suggesting that the bladder dysfunction associated with operational procedure might be the main cause of radiation-related bladder toxicity. Further clinical study is needed to verify it.

## Figures and Tables

**Figure 1:** Representative dose profiles of bladder in different filling states, underfilling, properly filling, or overfilling. The transverse plane (a) and sagittal plane (b) when bladder is underfilling; The transverse plane (c) and sagittal plane (d) when bladder is properly filling. The transverse plane (e) and sagittal plane (f) of bladder are over filling.

**Figure 2:** Relationship between the CTCAE grades and changes in bladder volume between the groups of post-op CRT and CRT alone. Post-op RT: post-operative CRT; RT: CRT.

**Figure 3:** (a) Relationship between the volume of bladder or bladder wall and the severity in CTCAE in 107 cases of cervical cancer. (b) The relationship between the volume of bladder or bladder wall exposed to radiation of 35 Gy or 40 Gy (V35 and V40) and the severity in CTCAE in 77 cases of stage I and II cervical cancer; BL: bladder; BW: bladder wall; V35 and V40: the volume covered by radiation dose of 35 Gy and 40 Gy, respectively.

**Table 1:** Characteristics for 107 patients with cervical cancer.

Item	Subcategory	No.	%
Age	>60	23	21.5
	40∼60	79	73.8
	<40	5	4.7
Pathological type	Squamous cell carcinoma	107	100.0
	Adenocarcinoma	0	0.0
	Adenosquamous carcinoma	0	0.0
FIGO stage	I	34	31.8
	II	43	40.1
	III/IV	30	28.0
Treatment modality	Surgery + post-op RT	65	60.7
	Concurrent chemo RT	38	35.5
	RT alone	4	3.7
Chemotherapy cycle	1∼2	22	20.6
	3∼4	43	40.2
	5∼6	28	26.2
	>6	10	9.3
RT technique	3D-CRT	0	0.0
	IMRT/VMAT	107	100.0
Dose for RT dose(Gy)	>60	7	6.5
	60	45	42.1
	50	46	43.0
	45/46	9	8.4
Bladder toxicity (CTCAE grade)	0	74	69.2
	1	23	21.5
	2	5	4.7
	3	5	4.7
	4	0	0.0
	5	0	0.0

RT: radiotherapy; Post-RT: post-operative CRT; Chemo-RT: CRT; 3D-CRT: 3-dimensional conformal radiotherapy; IMRT: intensify modulated radiotherapy; VMAT: volumetric modulated arc radiotherapy; CTCAE: common terminology criteria for adverse events.

**Table 2:** Comprehensive treatment of patients with different stages of cervical cancer.

Item	FIGO stage		
	I	II	III/IV
Case	34	43	30
Surgery (%)	97.06%	51.16%	33.33%
Frequency of RIC (%)	35.29%	39.53%	13.33%
Prescription dose (Gy)^*∗*^	50.06	55.20	59.49
Single dose (Gy)^*∗*^	2.00	2.19	2.30
Volume of CTV (cm^3^)^*∗*^	384.82	483.58	585.56
Volume of bladder (cm^3^)^*∗*^	325.56	310.56	315.70
Volume of bladder wall (cm^3^)^*∗*^	44.25	42.69	44.02
*D*_max_ (Gy)^*∗*^	54.52	59.16	63.99
D_mean_ (Gy)^*∗*^	41.03	42.05	44.02

^*∗*^Average value. RIC: radiation-induced cystitis; CTV: clinical tumor volume; *D*_max_: the maximal dose; D_mean_: the mean dose.

**Table 3:** Comparison of post-op radiotherapy and radiotherapy alone.

Item		Post-op RT	RT only
Case		65	42
CTCAE (%)	0	66.15%	73.81%
	1	20.00%	23.81%
	2	4.62%	2.38%
	3	9.23%	0.00%
Chemotherapy cycle^*∗*^		4.62	3.07
Prescription dose (Gy)^*∗*^		51.51	59.82
Single dose (Gy)^*∗*^		2.06	2.32
Volume of bladder (cm^3^)^*∗*^		329.96	296.17
*D*_max_ (Gy)^*∗*^		55.80	64.06
D_mean_ (Gy)^*∗*^		41.09	44.11

^*∗*^average value. CTCAE: common terminology criteria for adverse event; Post-op RT: post-operative CRT; RT: CRT; *D*_max_: the maximal dose; D_mean_: the mean dose.

**Table 4:** Comparison of the occurrence and nonoccurrence of radiotherapy toxicity in patients with stages I and II cervical cancer.

Item		CTCAE grade			
		0	1	2	3
Volume of bladder (cm^3^)^*∗*^		348.05	303.39	219.19	205.40
Volume of bladder wall (cm^3^)^*∗*^		47.09	41.07	34.85	29.81
Bladder	*D*_max_ (Gy)	57.28	57.85	53.13	56.19
	D_mean_ (Gy)	41.71	41.54	40.76	41.67
	V_35_ (cm^3^)	246.31	214.56	158.80	135.28
	V_40_ (cm^3^)	203.27	179.04	132.45	110.93
Bladder wall	*D*_max_ (Gy)	57.17	57.74	52.97	56.12
	D_mean_ (Gy)	44.33	43.77	42.33	43.29
	V_35_ (cm^3^)	45.88	43.17	35.36	32.58
	V_40_ (cm^3^)	41.43	38.81	31.65	29.07

^*∗*^: means average. CTCAE: common terminology criteria for adverse event; *D*_max_: the maximal dose; D_mean_: the mean dose; V_35_ and V_40_: the volume covered by radiation dose of 35 Gy and 40 Gy, respectively.

## Data Availability

The data used to support the findings of this study are available from the corresponding author upon request.
